The article "Emerging Role of Dendritic Cell Intervention in the Treatment of Inflammatory Bowel Disease" was published in 2022. Journal: Biomed Res Int.

# Emerging Role of Dendritic Cell Intervention in the Treatment of Inflammatory Bowel Disease

**DOI:** 10.1155/2022/7025634

**Published:** 2022-10-10

**Authors:** Donglei Sun, Chenyang Li, Shuang Chen, Xiaolan Zhang

**Affiliations:** ^1^Department of Gastroenterology, The Second Hospital of Hebei Medical University, Hebei Key Laboratory of Gastroenterology, Hebei Institute of Gastroenterology, Shijiazhuang, China; ^2^Department of Pediatrics and Department of Biomedical Science, Cedars Sinai Medical Center, Los Angeles, USA

## Abstract

Dendritic cells (DCs) are the most important antigen-presenting cells and are pivotal in initiating effective adaptive immune responses to induce immune tolerance and maintain immune homeostasis. Inflammatory bowel disease (IBD), including Crohn's disease and ulcerative colitis, is chronic, intestinal inflammatory and autoimmune disorder. DCs participate in IBD pathogenesis. This review is aimed at briefly discussing the role of DCs in IBD and the relationship between them and highlighting the prominent role of these cells in the treatment of these disorders.

## 1. Introduction

Inflammatory bowel disease (IBD) is a costly, severe, and chronic inflammation of the gastrointestinal tract. Some of its examples include Crohn's disease (CD) and ulcerative colitis (UC), which can be characterized by repeated phases of clinical relapses and remissions. However, the pathological mechanisms of IBD remain unclear. Innate and adaptive immune responses are known to play crucial roles in the pathogenesis and regulation of this illness [1]. Recent studies have focused on adaptive immune responses to explain the pathogenesis of IBD. In this regard, immunotherapy has emerged as a potentially attractive treatment target for IBD management.

Dendritic cells (DCs) are the most important antigen-presenting cells (APCs) of the immune system. These cells are implicated in IBD pathogenesis by genetics and microbial interactions and therefore may affect future therapeutic targets. In this narrative review, the role of DCs in IBD treatment is discussed.

## 2. Overview of IBD

IBD, including CD and UC, is a chronic form of inflammation of the GI tract [2] and is characterized by repeated phases of clinical relapses and remissions. This illness is a modern, incurable, autoimmune disease with low mortality.

### 2.1. The Pathogenesis of IBD

Genome-wide association studies in 100,000 patients with IBD revealed 200 loci associated with UC and CD [3, 4]. Most of the IBD-related loci are phenotypically dependent on intestinal microbes. Evidence of abnormal gut microbiota was documented in patients with IBD, but the potential pathogenic role of specific microorganisms remains unclear. More than 50% of IBD-related loci are associated with other autoimmune diseases, albeit with different effects [5]. Epidemiological data suggest an association between IBD and environmental factors such as smoking, drugs, geography, antibiotic use, social stress, and psychological elements [6].

### 2.2. Immunity and IBD

Although the aetiology of IBD has been studied extensively, its precise cause remains unclear. Innate immunity is thought to play an important role in the pathogenicity of IBD by initiating an adaptive immune response in response to specific antigens that are not yet understood [7]. Relevant immunological studies have focused on mucosal innate immune responses such as epithelial barrier integrity, innate microbial sensing, autophagy, and unfolded protein responses [8]. In patients with IBD, the behavior of cell-mediating innate immunity and the expression and function of Toll-like receptors (TLRs) and NOD proteins are significantly altered [9]. The immune system produces an excessive and abnormal immune response to the host microflora of genetically susceptible individuals, thereby causing IBD.

### 2.3. Treatment of IBD

Treatment modalities include corticosteroids, aminosalicylates, immunomodulators, antibiotics, probiotics, and a series of unique novel agents. The use of antitumor necrosis factor monoclonal antibody (infliximab, adalimumab), recombinant anti-inflammatory cytokines, and related gene therapy has been explored, and discussions regarding dietary supplementation and heparin treatment have commenced. Meanwhile, more and more new biological drugs that target different inflammatory pathways have been approved for the treatment of IBD: golimumab, vedolizumab, ustekinumab, certolizumab pegol, natalizumab, et al. Although the pathogenesis of this disease is diversified, no curative treatment scheme has been proposed so far.

## 3. Immunological Properties of DCs

DCs are the most important APCs with significant phenotypic heterogeneity and functional plasticity. These cells initiate effective adaptive immune responses to eliminate the invading pathogens, thereby inducing immune tolerance towards harmless components to maintain immune homeostasis, activate naïve T cells, and stimulate proliferation.

### 3.1. Subgroups of DCs

Human DCs originate from hematopoietic stem cells from two sources: myeloid dendritic cells generated from myeloid stem cells through the stimulation of granulocyte-macrophage colony-stimulating factor, which has a common myeloid progenitor with monocytes and neutrophils, and plasmacytoid dendritic cells (pDCs) generated from lymphoid stem cells and have a common myeloid progenitor with T cells and nature killing cells [10]. Recent studies revealed that these two DC subsets perform different functions in innate and adaptive immune responses [11].

### 3.2. DCs and Immunity

Most DCs exist as immature cells that typically express low levels of major histocompatibility complex II and costimulatory molecules and therefore are inclined to modulate T cell differentiation towards T helper 1 (Th1), T helper 2 (Th2), T helper 17 (Th17), or regulatory T (Treg) cell [12]. Th2 response is often associated with immune tolerance and can be used for the treatment of autoimmune diseases. Immature DCs express high levels of pattern recognition receptors (PRRs) to promote their maturation and activation.

### 3.3. DCs and Autoimmune Diseases

DCs could inhibit the immune response by producing reactive and regulatory T cells and change the quality of T cell activation and differentiation [13]. The pathogenesis of autoimmune diseases is closely linked with the breakdown of DC-mediated tolerance. DC ablation in mice under steady-state conditions resulted in a spontaneous autoimmune disease, indicating that these cells are essential in preventing autoimmunity and maintaining immune tolerance [14]. Newly developed immunotherapies are based on the tolerogenic potential of regulatory DCs for the treatment of autoimmune diseases. Treatment of cytokine cocktails including interleukin (IL)-10 or TNF-*α* generated DCs that can induce profound tolerance in the mouse models of collagen-induced arthritis, autoimmune thyroiditis, and other autoimmune diseases [15]. In addition, human intervention with DCs can regulate the immune response of the body and is of great practical significance for autoimmune diseases [16].

## 4. DCs and IBD

In IBD, the immune system fails to maintain immune tolerance and drives the development of proinflammatory T cells that control the progression of this disease [17]. DCs have emerged as central players whose genetic susceptibility impacts the mucosal immune system and regulates the response to gut microflora by acting as a bridge between innate and adaptive immune responses.

### 4.1. DC as a Sentry

DC precursors migrate to the mucosa in the GI tract, where they become sentinels and sensors of the immune system. DCs serve as sentinels because they sample their environment, and they are highly effective at capturing and processing antigens [18]. These cells also act as sensors that identify the nature of the sampled antigens and discriminate between potentially harmless and hazardous antigens because of their highly expressed PRR molecules [19]. Even in the presence of innate immune stress, DCs can still be activated. Recently, pDCs were found to be related to IBD onset and are highly enriched in the inflamed colon of patients with IBD; this enrichment correlates with disease severity [20, 21]. pDC depletion impaired the gut barrier function and led to severe colitis in a *Citrobacter rodentium*-induced colitis model [22]. Various molecules involved in the different steps of DC differentiation, maturation, migration, and activation have become potential therapeutic targets for combating autoimmune responses [23].

### 4.2. Different DC Subgroups and IBD

IBD patients in remission have slightly lower numbers of mDC compared with healthy control. In acute flare ups, IBD patients experience a significant drop of DC that correlates with disease activity [24]. The mucosa of CD patients is characterized by an increase in pDCs and, notably, most of these pDC clusters are highly expressed in IL-1*β* [25]. The proportion of cultured peripheral blood pDCs expressing CD40 and CD86 was significantly higher in patients with UC and CD compared to controls, and they also secreted significantly more tumor necrosis factor TNF-a, IL-6, and IL-8 [26]. Experiments on mice have shown that in equilibrium, pDCs can migrate to specific tissues, such as lymph glands or the intestine, under the control of chemokine receptors [27]. CD11c+ DCs, a subtype of cDCs, were reduced by more than 75% in CD patients with and without inflammation in the ileum compared to controls, while these noninflamed areas showed no significant injury or inflammation, suggesting that loss of DCs may be a precursor to subsequent injury [28]. In the presence of IL-15, all-trans RA induces the release of proinflammatory IL-12 and IL-23 from cDCs, promoting intestinal inflammation [29]. Several researchers have found that CD103 + cDCs in UC patients acquire a strong ability to drive Th1/Th2/Th17 cell responses, which is associated with increased expression of proinflammatory cytokines [30]. CD103+ cells were less frequent in active IBD intestinal tissue compared to controls [31]. The above evidence suggests a role for CDCs in IBD.

### 4.3. DC Activate Immunity of IBD

Intestinal DCs can successfully balance immune tolerance to nutrients and commensals and activate immunity against pathogens under normal circumstances [18, 32]. However, variations in this subtle balance are associated with the progression and development of IBD. The inflamed mucosa in patients with CD has a high number of proinflammatory 6-sulfo LacNAc (SLAN) +DCs, which can produce many cytokines from IL-23 to TNF-*α* that are involved in IBD pathogenesis. In healthy gut mucosa, DCs remain in a hypoactive, tolerogenic state; however, they change dramatically in IBD. Hart et al. demonstrated that only a minority of intestinal DCs are expressed TLR-2 or TLR-4 in healthy controls, and the expression of both types of TLRs is significantly enhanced in patients with CD and UC. A high level of the maturation/activation marker CD40 was expressed in freshly isolated DCs from the inflamed tissues of patients with CD. In addition, a large amount of colonic DCs produced IL-12 and IL-6 in CD but not in UC. Low numbers of CD103^+^ DCs were also found in the inflamed colon mucosa in CD. The mesenteric lymph nodes draining the inflamed tissues were found to contain a high number of CD11c^+^HLA-DR^+^ DCs [31]. The character of DC dysregulation in IBD is not restricted to the digestive tract because circulating DCs also show phenotypic and functional changes and exhibit a multihost profile. Patients with CD whose disease is restricted to different anatomical locations show a preferential migration capacity towards inflamed tissues [33], and this phenomenon may be correlated with the DC infiltrates found in target tissues.

### 4.4. DC and Gut Microecology in IBD

Enteric flora plays a vital role in the development of intestinal immune cells, including DCs. DCs distinguish pathogenic and commensal bacteria by using PRRs, including TLRs, C-type lectins such as mannose receptors, and the DC-specific intercellular adhesion molecule 3-grasping nonintegrin [34]. The microbial environment encounters an immature DC that matures to drive T cell differentiation towards Th1, Th2, or regulatory polarisation [35]. In response to specific microflora, DCs keeps a tolerant or protective immune response. The tolerogenic properties of DCs are potentially targeted for therapeutic settings. Emerging evidence states that the component changes of *Lactobacilli* cell surface can alter the immunoregulatory responses of DCs; this finding might open an avenue for a defined therapeutic pathway in the inflammatory diseases of the GI tract [36].

### 4.5. DC and Inflammatory Factors

Interferon (IFN)-*γ*-producing Th1 and IL-17-producing Th17 cells have been implicated in experimental colitis models and patients with IBD. The number of Th17 cells increases in inflamed patients with CD, and the IL-23 receptor variant associated with CD is damaged by the IL-23-induced Th17 effector function and works as a protective genetic variant [37]. Both are induced by a combination of IL-6 and TGF-*β* and promoted by IL-23 [38]. The involvement of Th17 cells and their signature cytokine IL-17A in intestinal inflammation has been extensively studied. Compared with that in a normal gut, high transcription levels of IL-17A were detected in the mucosa of CD and UC. Moreover, the inflamed IBD mucosa cultured *in vitro* produced higher levels of IL-17A than the control. The intrinsic involvement of receptor-interacting protein 2 (RIP2) in Th17 cell differentiation in a T cell appears as an essential mechanism for human chronic inflammatory diseases, including CD [39]. IL-23 in DCs is an essential component of the antimicrobial defence linking innate and adaptive immune responses. However, excessive or inappropriate amounts of IL-23 in DCs can result in the development of proinflammatory T cell responses, including the increased proliferation of effector T cells, the decreased differentiation of FoxP3-positive regulatory T cells, and the appearance of IL-17 and IFN-*γ*-producing cells associated with chronic intestinal inflammation. By contrast, IL-23R polymorphism is associated with the risk of protection against IBD, and its functional characteristics lead to a reduction in T cell activation [40, 41]. MiR-10a, which is highly expressed in intestine DCs, regulates IBD pathogenesis by inhibiting the expression of IL-12/IL-23 p40 and NOD2 in DC and the functions of Th1 and Th17 cells in IBD [42].

## 5. DC-Related Intervention in the Therapies of IBD

Given the unique characteristics of DCs, which are found at the junction between innate and secondary antigen-specific immune responses, these cells can be used as a target for clinical intervention in patients with IBD. Different DC subgroups use different transcription factors and, therefore, can be applied as different immunomodulatory targets.

### 5.1. DC and TL1A in IBD

Some DC processes associated with IBD genetic susceptibility have been identified as potential therapeutic targets. For example, blocking the interaction between DCs and T cells can weaken the vital action of IL-23/IL-17 inflammatory pathways in IBD pathogenesis. Activated DCs express the tumor necrosis factor cytokine 1A (TL1A), which interacts with the death receptor (DR) 3 on the lymphocyte. Therefore, the modulation of TL1A-DR3 interaction may be a potential therapeutic target in several autoimmune diseases. Given that TL1A expression is increased in CD tissues, anti-TL1A antibodies can prevent the occurrence of colitis in mice. Spontaneous intestinal inflammation occurred in mice with overexpressed TL1A. Therefore, TL1A may be a feasible dendritic cell target in IBD. Anti-TL1A antibody could inhibit the activation of intestinal fibroblasts in the T cell transplantation model of chronic colitis and reduce the synthesis of collagen, thereby ameliorating intestinal inflammation and fibrosis. The mechanism may be related to the suppression of the TGF-1/Smad 3 signalling pathway [43].

### 5.2. DC and Pathway

B leukotriene receptor 1 (BLT1) signalling in DCs controls Th1 and Th17 differentiation and 2,4,6-trinitrobenzenesulfonic acid- (TNBS-) induced colitis pathogenesis by regulating the production of proinflammatory cytokines, including IL-6, TNF-*α*, and IL-12 [44]. BLT1 regulates inflammatory cytokine release through G*α*i *βγ* subunit-phospholipase C*β* (PLC*β*)-PKC pathway. Therefore, BLT1 antagonists can reduce the inflammatory cytokines produced by human peripheral blood DCs. These findings reveal the critical role of BLT1 in regulating adaptive immunity and TNBS-induced colitis and its potential as a drug target for adaptive immune-mediated IBD [45]. Rapamycin, an antibiotic that triggers autophagy by forming complexes with mTOR-inhibiting flavokawain B (FKB) 12, is commonly used to increase autophagy in cell culture. This drug has also been successfully applied to treat patients with severely refractory CD and has shown protective effects on mouse colitis models, thereby implying its promising utilization [46].

### 5.3. Other Interventions

Ghavami et al. [47] found that probiotics play an important role in DC immunomodulation by regulating the expression of costimulatory molecules, proinflammatory cytokines, and TLRs in DCs from patients with IBD. DCreg administered via vasoactive intestinal peptide (DC-VIP) injection could alleviate the clinical and histopathology severity of TNBS-induced colitis in mice and has been tested in different mouse colitis models treated with dexamethasone and 1*α*,25(OH)_2_D_3_ or pulsed with enterobacterial extract for colitis prevention [48]. Mesenchymal stem cells (MSCs) play useful roles in DSS-induced colitis through its Gal-3 dependence and its inhibition of DC inflammatory phenotype. Therefore, bone marrow MSC/DC-targeted therapy is an effective treatment for chronic colitis [49]. However, the effects of bone marrow MSCs on colitis DCs have not been detected. Therefore, further research must focus on MSCs on DC phenotype and the function of colon infiltration in the pathogenesis of colitis induced by DSS. Suppression of pDC migration to colonic isolated lymphoid follicles abrogates the development of colitis [21]. Anti-inflammatory effects of Saccharomyces boulardii mediated by mDCs from patients with CD and UC [50]. Removal or diversion of gut-homing DC as well as T-cells is likely to be critical in prevention of gut focused inflammation in IBD [51].

## 6. Conclusion

DCs play important roles in the development and progression of IBD. A DC-related intervention provides a promising direction for IBD treatment. DCs could produce multiple proinflammatory and anti-inflammatory cytokines in response to environmental factors in patients with IBD and the mouse models of colitis. However, the following questions remain unclear: what are the differences in DC properties and mechanisms in CD and UC? Are the altered DC properties restricted to any subset or are all the subsets equally affected? Noninflammatory mucosal areas in patients with IBD show a proinflammatory cytokine environment that does not translate locally into macroscopic inflammation. Addressing these questions in future studies may expand our current knowledge of GI-DC to develop new therapies for IBD. Much research is needed to utilize DCs for IBD treatment.
